# Development and Validation of Prediction Model for High Ovarian Response in *In Vitro* Fertilization-Embryo Transfer: A Longitudinal Study

**DOI:** 10.1155/2021/7822119

**Published:** 2021-10-16

**Authors:** Xinsha Tan, Honglin Xi, Jing Yang, Wenfeng Wang

**Affiliations:** ^1^Department of Reproductive Medical Center, Affiliated Renhe Hospital of China Three Gorges University, Yichang 443002, China; ^2^Department of Reproductive Medical Center, Renmin Hospital of Wuhan University, Wuhan 430060, China; ^3^School of Science, Shanghai Institute of Technology, Shanghai 201418, China; ^4^International Academy of Visual Art and Engineering, London E16 1AH, UK; ^5^Interscience Institute of Management and Technology, Bhubaneswar 752054, India

## Abstract

**Objective:**

To develop and validate a prediction model for high ovarian response in *in vitro* fertilization-embryo transfer (IVF-ET) cycles.

**Methods:**

Totally, 480 eligible outpatients with infertility who underwent IVF-ET were selected and randomly divided into the training set for developing the prediction model and the testing set for validating the model. Univariate and multivariate logistic regressions were carried out to explore the predictive factors of high ovarian response, and then, the prediction model was constructed. Nomogram was plotted for visualizing the model. Area under the receiver-operating characteristic (ROC) curve, Hosmer-Lemeshow test and calibration curve were used to evaluate the performance of the prediction model.

**Results:**

Antral follicle count (AFC), anti-Müllerian hormone (AMH) at menstrual cycle day 3 (MC3), and progesterone (P) level on human chorionic gonadotropin (HCG) day were identified as the independent predictors of high ovarian response. The value of area under the curve (AUC) for our multivariate model reached 0.958 (95% CI: 0.936-0.981) with the sensitivity of 0.916 (95% CI: 0.863-0.953) and the specificity of 0.911 (95% CI: 0.858-0.949), suggesting the good discrimination of the prediction model. The Hosmer-Lemeshow test and the calibration curve both suggested model's good calibration.

**Conclusion:**

The developed prediction model had good discrimination and accuracy via internal validation, which could help clinicians efficiently identify patients with high ovarian response, thereby improving the pregnancy rates and clinical outcomes in IVF-ET cycles. However, the conclusion needs to be confirmed by more related studies.

## 1. Introduction

With the rapid development of assisted reproductive technology (ART), *in vitro* fertilization-embryo transfer (IVF-ET) has become an important treatment for infertility [1]. Controlled ovarian hyperstimulation (COH) is a key step of IVF-ET, where gonadotropin (Gn) stimulates the development of multiple follicles and produces multiple mature oocytes, thereby improving pregnancy rates [2, 3]. However, it cannot be ignored that ovaries' overreaction to Gn could increase the risk of iatrogenic complication-ovarian hyperstimulation syndrome (OHSS) [4], which is characterized by an increase in ovarian volume and brings more severe and even fatal infertility. Therefore, it is still necessary to identify the risk of OHSS in IVF-ET for patients.

High ovarian response, defined as excessive ovarian response, is reported as an adverse effect of IVF-ET [5]. It is mainly due to changes in the systemic stress state led by the recruitment and development of multiple follicles and abnormally high steroid substances [5]. Hormone level is higher in patients with high ovarian response, which is not conducive to endometrial receptivity and embryo implantation, thereby increasing the incidence of ovarian hyperstimulation syndrome (OHSS) [6]. In view of this, it is of great clinical significance to find predictors for high ovarian response, which may decrease the risk of OHSS, improve pregnancy rates, and optimize pregnancy outcomes.

Previous studies verified that anti-Müllerian hormone (AMH) and antral follicle count (AFC) were the effective predictors of high ovarian response [7–12]. In the study of Oehninger et al., female age and follicle-stimulating hormone (FSH) were also found to be the predictors of high ovarian response [13]. To our knowledge, most studies focused on the predictive factors of poor ovarian response, and few studies have been done on predictive factors of high ovarian response. Not only that, a complete predictive system on high ovarian response has not been established yet, and there are only some researches of individual indicators, which was not accurate for predicting high ovarian response. Hence, this study was to explore the independent predictors of high ovarian response in patients undergoing IVF-ET and set out to develop a model for predicting the risk of high ovarian response and perform internal validation. We believed that the results will provide better guidance to the clinical use of a reasonable COH protocol, thereby improving pregnancy rates and clinical outcomes in IVF-ET cycles.

## 2. Methods

### 2.1. Collection of the Data

A longitudinal study of 1,142 outpatients with infertility who underwent IVF-ET at the Affiliated Renhe Hospital of China Three Gorges University from January 2018 to December 2019 was consecutively selected. The patients were divided into high ovarian response group (>15 oocytes retrieved) and normal ovarian response group (4-15 oocytes retrieved) [9, 14]. The inclusion criteria were as follows: (1) patients aged 20-40 years with normal menstrual cycles (21-35 days); (2) patients undergoing IVF-ET; (3) patients with complete clinical data. Patients were excluded if met any of the following criteria: (1) patients who were diagnosed with polycystic ovary syndrome (PCOS) according to Rotterdam criteria; (2) patients who had primary ovarian insufficiency; (3) patients who had ovarian-related surgery before (such as laparoscopic ovarian drilling, ovarian dissection for endometriosis, unilateral oophorectomy); (4) patients who had hormonal contraceptives before study cycle; (5) patients who had taken other investigational drugs or was participating in other clinical studies within 1 month before study enrolment; (6) physician considered patients who were inappropriate to participate in the clinical investigator.

The study was approved by the Ethics Committee of Affiliated Renhe Hospital of China Three Gorges University with the number of 2020K05. Signed informed consent was obtained from all patients before enrollment.

Gonadotropin-releasing hormone (GnRH) agonist was subcutaneously injected on the 21st day of menstruation to downregulate the function of pituitary gland. After 14 days, COH was initiated with the appropriate amount of Gn (150-300 U/d) according to age, body mass index (BMI), and baseline FSH. The development of follicles was monitored by ultrasound. When 1-2 follicles were ≥18 mm in diameter, or 2-3 were ≥17 mm in diameter, 10,000 U of human chorionic gonadotropin (HCG) was injected. Oocytes were retrieved 36 h after HCG injection, and embryo transfer was performed 3-5 days after retrieval, after which 80 mg of progesterone (P) was intramuscularly injected daily as luteal support. A positive serum HCG pregnancy test after 14 days was defined as biochemical pregnancy, and ultrasound confirmation of a gestational sac or heartbeat (fetal pole) 35 days after transfer was diagnosed as clinical pregnancy.

### 2.2. Analytic Methods

Baseline characteristics of patients were collected in our study, of which categorical variables included smoking history, type of infertility, and pregnancy history; continuous variables contained age, BMI, age at menarche, mean menstrual cycle, and duration of infertility; AFC, endometrial thickness, luteinizing hormone (LH) level, estradiol (E2) level, P level, FSH level, and AMH level on menstrual cycle day 3 (MC3); dosing days, initial dose, and total dose of Gn; endometrial thickness and hormone levels on the day of HCG injection. AFC was assessed by transvaginal sonography at MC3; endometrial thickness was observed on the day of injection of HCG; LH was defined as a hormone secreted by basophils in the anterior pituitary gland; E2 was a steroidal estrogen with the normal value of follicular stage (94-433 pmol/L), the normal value of luteal phase (499-1580 pmol/L), and the normal value during ovulation (704-1580 pmol/L); P was defined as main progesterone with biological activity secreted by the ovary; FSH was a hormone secreted by basophils in the anterior pituitary gland that promoted follicle maturation; AMH was defined as a hormone secreted by follicles in the predeveloping chambers or small chambers of the ovary. In addition, dosing days, initial dose, and total dose of Gn, endometrial thickness, and hormone level on the day of HCG injection were collected for analyzing the predictive factors of high ovarian response.

The measurement data was tested by the Kolmogorov-Smirnov test for normality. Normally distributed continuous variables were expressed as mean ± standard deviation (Mean ± SD), and Student's *t* test was used for comparison between groups; continuous variables with skewed distribution were expressed as median and quartile [*M* (*Q*_1_, *Q*_3_)], and the Mann-Whitney *U* test was applied for comparison. Categorical variables were expressed as number of cases and constituent ratio [*n* (%)], and the Chi-square test and Fisher's exact test were used for comparison. The two-sided test was performed for all statistical analyses, and *P* < 0.05 was considered statistically significant. All statistical analysis was performed by using SAS 9.4 and R 4.0.2 (model validation and drawing) statistical software. Prediction models were constructed by adopting SAS 9.4 (Logistic model) and Python 3.7 [Broad Learning System (BLS) model] software.

In the present study, the population was randomly divided into training set for developing the prediction logistic model and BLS model, and testing set for validating the models at the ratio of 7 : 3. Univariate and multivariate logistic regressions were carried out to explore the predictive factors of high ovarian response, and then, the prediction model was constructed. Nomogram was plotted for visualizing the model. Area under the receiver-operating characteristic (ROC) curve, the Hosmer-Lemeshow test, and calibration curve were used to evaluate the performance of the prediction model. The Youden index was used to calculate the cutoff point, which was identified as the cutoff point at a high risk for high ovarian response. Then, the comparison of predictive power was carried out between the logistic model and BLS model for high ovarian response.

## 3. Results

### 3.1. Patient Characteristics

Among the total 1,142 outpatients, patients who were over 40 years old (*n* = 63) were pretreated with hormonal contraceptives before study cycle (*n* = 54), had ovarian-related surgery before (*n* = 47), had primary ovarian insufficiency (*n* = 28), were diagnosed with PCOS according to Rotterdam criteria (*n* = 196), had low ovarian response (*n* = 264), or had missing information of age and BMI (*n* = 10) were excluded. 480 eligible outpatients were enrolled with 336 patients in the training set and 144 in the testing set eventually. Then, the patients were divided into the high response group (HR group, *n* = 239) and the normal response group (NR group, *n* = 241). The mean age was 31.36 ± 3.79 years, and the mean age at menarche was 13.16 ± 1.22 years. Only 6 (1.25%) patients reported the history of active smoking, 75 (15.63%) had the history of passive smoking, and the remaining 399 (83.13%) had no smoking history. The mean menstrual cycle was 29.23 ± 2.04 days, and the median duration of infertility was 3.00 (1.00, 4.00) years.  Table 1 gives an overview of baseline characteristics of all patients. No significant differences were observed between the training set and the testing set in all variables (all *P* > 0.05).

### 3.2. Risk Factor Selection

The results of Table 2 suggested that age, mean menstrual cycle, AFC, P at MC3, FSH at MC3, AMH at MC3, initial dose of Gn, total dose of Gn, LH on HCG day, E2 on HCG day, and P level on HCG day in the high response group were significantly different from those in the normal response group (all *P* < 0.05), which could be considered as potential predictors and included in the multivariate analysis (Table 3).

### 3.3. Development and Visualization of the Prediction Model

To identify predictors for high ovarian response in IVF-ET, the multivariate logistic regression was performed. The results indicated that AFC, AMH at MC3, and P level on HCG day were independently associated with high ovarian response. For each additional AFC, the risk of high ovarian response increased by 0.671-fold (95% CI: 1.453-1.921, *P* < 0.001). For every 1 ng/mL increase in AMH at MC3, the risk of high response increased by 0.874-fold (95% CI: 1.404-2.502, *P* < 0.001). Besides, the risk rose by 0.950-fold for every 1 nmol/L increase in P on the day of HCG injection (95% CI: 1.141-3.331, *P* = 0.015) (Table 4). Then, the predicted risk of high ovarian response was calculated as follows: Ln (*P*_*HR*_/(1 − *P*_*HR*_)) = −11.094 + AFC∗0.513 + AMH at MC3∗0.628 + P on HCG day∗0.668 (*P*_*HR*_ represented the probability of high ovarian response).

To visualize our model, the nomogram was plotted (Figure 1). For example, we randomly chose a patient whose P at HCG day was 0.53 nmol/L, AMH at MC3 was 3.6 ng/mL, and AFC was 18. The total point was 134, and the predicted probability of high ovarian response was 0.682 (Figure 2), which was higher than optimum cutoff point 0.491 (Table 5) and indicated a higher incidence of high ovarian response.

### 3.4. Validation of the Prediction Model

According to the ROC analysis, the AUC values for AFC, AMH at MC3, and P level on HCG day were 0.937 (95% CI: 0.911-0.963), 0.905 (95% CI: 0.871-0.939), and 0.692 (95% CI: 0.636-0.749), respectively (Table 5, Figure 3). For the multivariate model combining the above predictors, the AUC reached 0.958 (95% CI: 0.936-0.981) with the sensitivity of 0.916 (95% CI: 0.863-0.953) and the specificity of 0.911 (95% CI: 0.858-0.949), revealing a better performance on the prediction of high ovarian response (Figures 3 and 4). Additionally, the AUC of the testing set was 0.950 (0.918-0.983) with the sensitivity of 0.875 (0.799-0.951) and the specificity of 0.875 (0.799-0.951) (Table 6, Figure 4), which confirmed the good discrimination of the model. The Hosmer-Lemeshow test showed the good calibration of the model (training set: *χ*^2^ = 0.046, *P* = 0.829; testing set: *χ*^2^ = 7.497, *P* = 0.484). The calibration curve also confirmed the good calibration of our model (Figure 4).

### 3.5. Comparison for the Prediction Models

As a novel neural network model based on random vector functional-link neural network (RVFLNN), BLS is suitable for processing relatively simple data and has a faster learning speed [15]. Therefore, we constructed a BLS model with 4 feature nodes per window, 5 feature node windows, 9 enhancement nodes, incremental steps (3), number of reinforcement nodes (50), coefficient of compressibility (0.7), and regularization coefficient (2^−30^) and compared its predictive power with the logistic model. The predictors of our logistic model were put into the BLS model to assess the predictive power. The results showed that the AUC and accuracy of the BLS model were inferior to the logistic model (Table 7). It was indicated that the BLS model may be not suitable for simple data which included only three variables. The ROC curves for the training set and the testing set of the BLS model are displayed in Figure 5.

## 4. Discussion

High ovarian response can induce the risk of OHSS, leading to the increased discomfort in patients and even reducing prospects for pregnancy [16]. Up to 30% of cases with mild or moderate OHSS and 3-8% with severe OHSS were reported in IVF-ET cycles [17]. In this study, we aimed to develop a prediction model to predict the risk of high ovarian response in patients undergoing IVF-ET. Our results suggested that AFC, AMH at MC3, and P level on HCG day were the three effective predictors for high ovarian response in IVF-ET cycles. What is more, a combined prediction model with good performance was developed and validated: Ln (*P*_*HR*_/(1 − *P*_*HR*_)) = −11.094 + AFC∗0.513 + AMH at MC3∗0.628 + P on HCG day∗0.668 (*P*_*HR*_ represented the probability of high ovarian response). Simultaneously, we plotted a nomogram for visualizing our model; the AUC value of the combined prediction model reached 0.958, which suggested the good discrimination of the model, and the internal validation confirmed the accuracy and feasibility of the model. Further, the Hosmer-Lemeshow test and the calibration curve showed the good calibration of our model. We believed that the finding could make it easier for clinicians to predict high ovarian response in IVF-ET cycles and develop individualized treatment strategies for patients, thereby reducing the incidence rates of OHSS and improving pregnancy rates and clinical outcomes.

In our study, both AFC and basal AMH were independently associated with high ovarian response, which was consistent with the results of previous researches [9, 18–20]. Aflatoonian et al. reported that AMH and AFC were considered as the accurate and reliable predictors of high ovarian response to COH and could identify the patients who had an increased risk of OHSS before stimulation [18]. The reason may be that AMH concentration correlates significantly with the number of sinusoidal follicles in the ovary before ovulation and the number of oocytes collected after treatment, and patients with high ovarian response have higher AMH concentration compared with patients with normal ovarian response. Not only that, AMH was regarded as an excellent predictor of high ovarian response and could identify the risk of OHSS better than AFC, which may be due to the fact that AMH has more stable periodicity and is less susceptible to exogenous steroid hormones; moreover, AFC requires skilled ultrasound operators to carefully identify, measure, and count ovarian eggs, probably resulting in more interobserver variability in AFC [7, 18, 21–25]. However, few studies have analyzed the association between P level on HCG day and high ovarian response. In a retrospective study, P level at the first day of stimulation was recorded as a potential predictor, but no statistical significance was found [26]. Studies have shown that P level on the day of HCG administration varies among different ovarian responders [27–29]. Whether the P level can affect pregnancy rates and IVF-ET outcomes remains to be verified in further research. More importantly, our study showed that the model including all predictors had a more accurate predictive power for high ovarian response than the one containing independent predictors. The possible explanation may be that considering only one factor to predict the probability of high ovarian response and ignoring the existence of other factors may reduce predictive ability and increase the error brought by independent factor. However, our conclusion needs to be confirmed by more related studies.

The strengths of the study should be noted. We identified predictors for high ovarian response in IVF-ET and developed a prediction model with more accurate predictive power, which could help clinicians efficiently identify patients at a risk of high ovarian response and individualize treatment for these patients. However, there were also some limitations in our study. Firstly, women aged 20-40 years were enrolled in our study, which may be considered as nonrepresentative samples. This is mainly due to the fact that women of this age group have better fertility with more ideal stimulation effect. A wider range of ages could be considered in the future research to improve the universality of the model. In addition, small sample size and lack of external validation may affect the general applicability of our model. A multicenter study with large sample size and external validation is required to improve the accuracy and reliability of the model.

## 5. Conclusion

The developed prediction model had good discrimination and accuracy through the internal validation, which could help clinicians identify patients with high ovarian response, thereby improving pregnancy rates and clinical outcomes in IVF-ET cycles.

## Figures and Tables

**Figure 1:** Logistic nomogram for predicting high ovarian response.

**Figure 2:** Example for the application of the nomogram.

**Figure 3:** ROC curves for single factor and the combined prediction model.

**Figure 4:** ROC (a) and calibration curves (b) for the training set and the testing set of the logistic model.

**Figure 5:** ROC curves for the training set and the testing set of the BLS model.

**Table 1:** Baseline characteristics of study population.

Variables, *n* (%)	Total (*n* = 480)	Group		Statistic	*P*
		Training set (*n* = 336)	Testing set (*n* = 144)		
Age, years, mean ± SD	31.36 ± 3.79	31.26 ± 3.79	31.59 ± 3.77	*t* = −0.86	0.389
BMI, kg/m^2^, mean ± SD	22.08 ± 2.97	21.99 ± 2.97	22.29 ± 2.97	*t* = −1.00	0.317
Smoking history, *n* (%)				*Z* = −0.933	0.351
Active smoking	6 (1.25)	5 (1.49)	1 (0.69)		
Passive smoking	75 (15.63)	48 (14.29)	27 (18.75)		
No	399 (83.13)	283 (84.23)	116 (80.56)		
Type of infertility, *n* (%)				*χ* ^2^ = 2.887	0.089
Primary	174 (36.25)	130 (38.69)	44 (30.56)		
Secondary	306 (63.75)	206 (61.31)	100 (69.44)		
Pregnancy history, *n* (%)				*χ* ^2^ = 2.796	0.094
No	177 (36.88)	132 (39.29)	45 (31.25)		
Yes	303 (63.13)	204 (60.71)	99 (68.75)		
Age at menarche, years, mean ± SD	13.16 ± 1.22	13.14 ± 1.20	13.22 ± 1.26	*t* = −0.60	0.551
Mean menstrual cycle, days, mean ± SD	29.23 ± 2.04	29.28 ± 2.04	29.10 ± 2.06	*t* = 0.87	0.385
Duration of infertility, years, *M* (*Q*_1_, *Q*_3_)	3.00 (1.00, 4.00)	3.00 (2.00, 4.00)	3.00 (1.00, 4.50)	*Z* = −0.544	0.586
AFC, *M* (*Q*_1_, *Q*_3_)	15.00 (12.00, 20.00)	15.00 (12.00, 19.00)	15.00 (12.00, 20.00)	*Z* = 0.293	0.770
LH, mu/mL, *M* (*Q*_1_, *Q*_3_)	4.79 (3.61, 6.24)	4.79 (3.54, 6.02)	4.75 (3.72, 6.34)	*Z* = 1.248	0.212
MC3					
E2, pmol/L, *M* (*Q*_1_, *Q*_3_)	36.18 (25.95, 46.42)	36.16 (26.26, 46.38)	36.60 (25.57, 46.49)	*Z* = −0.521	0.602
P, nmol/L, *M* (*Q*_1_, *Q*_3_)	0.39 (0.26, 0.59)	0.40 (0.26, 0.59)	0.35 (0.25, 0.56)	*Z* = −1.223	0.221
FSH, U/L, mean ± SD	6.50 ± 1.60	6.56 ± 1.69	6.36 ± 1.35	*t* = 1.33	0.186
AMH, ng/ml, *M* (*Q*_1_, *Q*_3_)	3.71 (2.46, 5.27)	3.68 (2.46, 5.25)	3.75 (2.46, 5.33)	*Z* = −0.108	0.914
Endometrial thickness, mm, mean ± SD	10.05 ± 2.09	10.09 ± 2.10	9.96 ± 2.08	*t* = 0.63	0.526
Group				*χ* ^2^ = 0.004	0.952
Normal response	241 (50.21)	169 (50.30)	72 (50.00)		
High response	239 (49.79)	167 (49.70)	72 (50.00)		

BMI: body mass index; AFC: antral follicle count; LH: luteinizing hormone; MC3: menstrual cycle day 3; E2: estradiol; P: progesterone; FSH: follicle-stimulating hormone; AMH: anti-Müllerian hormone; Mean ± SD: mean ± standard deviation; *M* (*Q*_1_, *Q*_3_): median and quartile; *χ*^2^: measured the degree of correlation between two categorical variables; *t*: compared the difference between the two groups; *Z*: represented the rank sum test for the comparison of two samples.

**Table 2:** Difference analysis for the potential predictors of ovarian response in IVF-ET.

Variables, *n* (%)		Total (*n* = 336)	HR group (*n* = 167)	NR group (*n* = 169)	Statistic	*P*
Baseline	Age, years, mean ± SD	31.26 ± 3.79	30.73 ± 3.67	31.79 ± 3.85	*t* = −2.588	0.010
	Smoking history				—	0.686
	Active smoking	5 (1.49)	3 (1.80)	2 (1.18)		
	Passive smoking	48 (14.29)	26 (15.57)	22 (13.02)		
	No	283 (84.23)	138 (82.63)	145 (85.80)		
	Type of infertility				*χ* ^2^ = 3.530	0.060
	Primary	130 (38.69)	73 (43.71)	57 (33.73)		
	Secondary	206 (61.31)	94 (56.29)	112 (66.27)		
	Pregnancy history				*χ* ^2^ = 1.452	0.228
	No	132 (39.29)	71 (42.51)	61 (36.09)		
	Yes	204 (60.71)	96 (57.49)	108 (63.91)		
	BMI, kg/m^2^, mean ± SD	21.99 ± 2.97	22.05 ± 3.06	21.94 ± 2.88	*t* = 0.340	0.734
	Age at menarche, years, mean ± SD	13.14 ± 1.20	13.06 ± 1.11	13.22 ± 1.29	*t* = −1.259	0.209
	Mean menstrual cycle, days, mean ± SD	29.28 ± 2.04	29.62 ± 2.15	28.94 ± 1.87	*t* = 3.091	0.002
	Duration of infertility, years, *M* (*Q*_1_, *Q*_3_)	3.00 (2.00, 4.00)	3.00 (2.00, 5.00)	3.00 (1.00, 4.00)	*Z* = 1.430	0.153
	AFC, *M* (*Q*_1_, *Q*_3_)	15.00 (12.00, 19.00)	19.00 (16.00, 22.00)	12.00 (10.00, 14.00)	*Z* = 13.879	<0.001
MC3	LH, mu/ml, *M* (*Q*_1_, *Q*_3_)	4.79 (3.54, 6.02)	4.87 (3.61, 6.01)	4.71 (3.32, 6.04)	*Z* = 0.274	0.784
	E2, pmol/L, *M* (*Q*_1_, *Q*_3_)	36.16 (26.26, 46.38)	35.23 (23.22, 45.70)	37.56 (27.80, 47.44)	*Z* = −1.903	0.057
	P, nmol/L, *M* (*Q*_1_, *Q*_3_)	0.40 (0.26, 0.59)	0.46 (0.31, 0.66)	0.32 (0.22, 0.48)	*Z* = 4.626	<0.001
	FSH, U/L, mean ± SD	6.56 ± 1.69	6.34 ± 1.65	6.77 ± 1.71	*t* = −2.304	0.022
	AMH, ng/ml, *M* (*Q*_1_, *Q*_3_)	3.68 (2.46, 5.25)	5.20 (4.19, 6.17)	2.69 (2.01, 3.34)	*t* = 14.188	<0.001
	Endometrial thickness, mm, mean ± SD	10.09 ± 2.10	10.18 ± 2.07	10.00 ± 2.13	*t* = 0.798	0.425
HCG day	Dosing days of Gn, days, mean ± SD	12.13 ± 2.63	12.26 ± 2.55	12.01 ± 2.71	*t* = 0.86	0.393
	Initial dose of Gn, IU, mean ± SD	217.82 ± 54.94	208.80 ± 50.98	226.70 ± 57.37	*t* = −3.02	0.003
	Total dose of Gn, IU, mean ± SD	2861.99 ± 919.51	2753.70 ± 821.50	2969.00 ± 998.00	*t* = −2.16	0.032
	Endometrial thickness, mm, mean ± SD	11.10 ± 2.32	11.31 ± 2.34	10.89 ± 2.28	*t* = 1.67	0.095
	LH, mu/mL, *M* (*Q*_1_, *Q*_3_)	0.95 (0.55, 1.87)	0.84 (0.53, 1.42)	1.15 (0.55, 2.14)	*Z* = −2.161	0.031
	E2, pmol/L, *M* (*Q*_1_, *Q*_3_)	2986.00 (2074.86, 4857.50)	4403.00 (2811.00, 6000.00)	2405.00 (1657.00, 3483.00)	*Z* = 8.737	<0.001
	P, nmol/L, *M* (*Q*_1_, *Q*_3_)	0.95 (0.67, 1.32)	1.16 (0.82, 1.56)	0.81 (0.57, 1.12)	*Z* = 6.089	<0.001

HR group: high response group; NR group: normal response group; BMI: body mass index; AFC: antral follicle count; MC3: menstrual cycle day 3; LH: luteinizing hormone; E2: estradiol; P: progesterone; FSH: follicle-stimulating hormone; AMH: anti-Müllerian hormone; HCG: human chorionic gonadotropin; Gn: gonadotropin; Mean ± SD: mean ± standard deviation; *M* (*Q*_1_, *Q*_3_): median and quartile; *χ*^2^: measured the degree of correlation between two categorical variables; *t*: compared the difference between the two groups; *Z*: represented the rank sum test for the comparison of two samples.

**Table 3:** Univariate analysis for the potential predictors of high ovarian response in IVF-ET.

Variables, *n* (%)	*β*	S.E	Wald	*P*	OR	95% CI	
						Lower	Upper
Age	-0.075	0.030	6.489	0.011	0.927	0.875	0.983
BMI	0.013	0.037	0.116	0.734	1.013	0.942	1.088
Smoking history							
No					Ref		
Active smoking	0.455	0.921	0.244	0.621	1.576	0.259	9.576
Passive smoking	0.217	0.313	0.478	0.489	1.242	0.672	2.294
Type of infertility							
Primary					Ref		
Secondary	-0.423	0.225	3.515	0.061	0.655	0.421	1.019
Pregnancy history							
No					Ref		
Yes	-0.270	0.224	1.449	0.229	0.764	0.492	1.185
Age at menarche	-0.115	0.092	1.572	0.210	0.891	0.745	1.067
Mean menstrual cycle	0.172	0.057	8.918	0.003	1.187	1.061	1.329
Duration of infertility	0.056	0.047	1.390	0.238	1.057	0.964	1.159
AFC	0.641	0.070	84.345	<0.001	1.898	1.655	2.176
LH at MC3	0.010	0.025	0.167	0.683	1.010	0.962	1.061
E2 at MC3	-0.002	0.004	0.367	0.545	0.998	0.991	1.005
P at MC3	0.143	0.121	1.389	0.238	1.154	0.909	1.464
FSH at MC3	-0.151	0.067	5.139	0.023	0.859	0.754	0.980
AMH at MC3	1.207	0.128	89.114	<0.001	3.345	2.603	4.298
Endometrial thickness at MC3	0.042	0.052	0.637	0.425	1.043	0.941	1.155
Dosing days of Gn	0.036	0.042	0.729	0.393	1.036	0.955	1.125
Initial dose of Gn	-0.006	0.002	8.675	0.003	0.994	0.990	0.998
Total dose of Gn	-0.000	0.000	4.513	0.034	1.000	0.999	1.000
Endometrial thickness on HCG day	0.079	0.048	2.774	0.096	1.083	0.986	1.189
LH on HCG day	-0.199	0.077	6.743	0.009	0.820	0.705	0.952
E2 on HCG day	0.001	0.000	56.290	<0.001	1.001	1.000	1.001
P on HCG day	0.679	0.197	11.898	<0.001	1.971	1.340	2.898
FSH on HCG day	0.018	0.019	0.911	0.340	1.018	0.981	1.057

BMI: body mass index; AFC: antral follicle count; MC3: menstrual cycle day 3; LH: luteinizing hormone; E2: estradiol; P: progesterone; FSH: follicle-stimulating hormone; AMH: anti-Müllerian hormone; HCG: human chorionic gonadotropin; Gn: gonadotropin; S.E: standard error; OR: odds ratio; CI: confidence interval.

**Table 4:** Multivariate analysis for the predictors of high ovarian response in IVF-ET.

Variables, *n* (%)	*β*	S.E	Wald	*P*	OR	95% CI	
						Lower limit	Upper limit
Constant	-11.094	1.219	82.822	<0.001			
AFC	0.513	0.071	51.996	<0.001	1.671	1.453	1.921
AMH at MC3	0.628	0.148	18.151	<0.001	1.874	1.404	2.502
P on HCG day	0.668	0.273	5.974	0.015	1.950	1.141	3.331

AFC: antral follicle count; AMH: anti-Müllerian hormone; MC3: menstrual cycle day 3; P: progesterone; HCG: human chorionic gonadotropin. S.E: standard error; OR: odds ratio; CI: confidence interval.

**Table 5:** Performance comparison of predictors for high ovarian response by ROC analysis.

Predictors	AUC (95% CI)	Cut-off	Sensitivity (95% CI)	Specificity (95% CI)	*Z*	*P*
Combination	0.958 (0.936-0.981)	0.491	0.916 (0.874-0.958)	0.911 (0.868-0.954)	—	
AFC	0.937 (0.911-0.963)	0.603	0.868 (0.817-0.920)	0.890 (0.841-0.942)	2.707	0.007
AMH at MC3	0.905 (0.871-0.939)	0.525	0.820 (0.762-0.879)	0.911 (0.868-0.954)	3.905	<0.001
P on HCG day	0.692 (0.636-0.749)	0.484	0.611 (0.537-0.685)	0.662 (0.588-0.767)	8.899	<0.001

AMH: anti-Müllerian hormone; AFC: antral follicle count; MC3: menstrual cycle day 3; P: progesterone; HCG: human chorionic gonadotropin; CI: confidence interval.

**Table 6:** Predictive value of the logistic model for high ovarian response.

Variables	Data set	
	Training set	Testing set
AUC (95% CI)	0.958 (0.936-0.981)	0.950 (0.918-0.983)
Accuracy (95% CI)	0.914 (0.884-0.944)	0.875 (0.821-0.929)
Sensitivity (95% CI)	0.916 (0.874-0.958)	0.875 (0.799-0.951)
Specificity (95% CI)	0.911 (0.868-0.954)	0.875 (0.799-0.951)
PPV (95% CI)	0.911 (0.868-0.954)	0.875 (0.799-0.951)
NPV (95% CI)	0.917 (0.875-0.958)	0.875 (0.799-0.951)

AUC: area under the curve; PPV: positive predictive value; NPV: negative predictive value; CI: confidence interval.

**Table 7:** The predictive value of the BLS model for high ovarian response.

Variables	Training set	Testing set
AUC (95% CI)	0.692 (0.636-0.748)	0.706 (0.622-0.791)
Accuracy (95% CI)	0.613 (0.561-0.666)	0.625 (0.546-0.704)
Sensitivity (95% CI)	0.964 (0.936-0.992)	0.958 (0.912-1.000)
Specificity (95% CI)	0.266 (0.200-0.333)	0.292 (0.187-0.397)
PPV (95% CI)	0.565 (0.507-0.324)	0.575 (0.487-0.380)
NPV (95% CI)	0.882 (0.794-0.971)	0.875 (0.743-1.000)

AUC: area under the curve; PPV: positive predictive value; NPV: negative predictive value; CI: confidence interval.

## Data Availability

All the data utilized to support the theory and models of the present study are available from the corresponding authors upon request.

## References

[1] Pereira N., Petrini A. C., Zhou Z. N., Lekovich J. P., Kligman I., Rosenwaks Z. (2016). Pretreatment of normal responders in fresh in vitro fertilization cycles: a comparison of transdermal estradiol and oral contraceptive pills. *Clinical and Experimental Reproductive Medicine*.

[2] Duan L., Bao S., Li K., Teng X., Hong L., Zhao X. (2017). Comparing the long-acting and short-acting forms of gonadotropin-releasing hormone agonists in the long protocol of IVF/ICSI cycles: a retrospective study. *The Journal of Obstetrics and Gynaecology Research*.

[3] Gao M., Jiang X., Li B. (2019). Intrauterine injection of human chorionic gonadotropin before embryo transfer can improve in vitro fertilization-embryo transfer outcomes: a meta-analysis of randomized controlled trials. *Fertility and Sterility*.

[4] Nelson S. M. (2017). Prevention and management of ovarian hyperstimulation syndrome. *Thrombosis Research*.

[5] Sunkara S. K., Rittenberg V., Raine-Fenning N., Bhattacharya S., Zamora J., Coomarasamy A. (2011). Association between the number of eggs and live birth in IVF treatment: an analysis of 400 135 treatment cycles. *Human Reproduction*.

[6] Kawwass J. F., Kissin D. M., Kulkarni A. D. (2015). Safety of assisted reproductive technology in the United States, 2000-2011. *JAMA*.

[7] Bedenk J., Vrtačnik-Bokal E., Virant-Klun I. (2020). The role of anti-Müllerian hormone (AMH) in ovarian disease and infertility. *Journal of Assisted Reproduction and Genetics*.

[8] Broekmans F. J., Kwee J., Hendriks D. J., Mol B. W., Lambalk C. B. (2006). A systematic review of tests predicting ovarian reserve and IVF outcome. *Human Reproduction Update*.

[9] Huang J., Lin J., Gao H. (2019). Anti-Müllerian hormone for the prediction of ovarian response in progestin-primed ovarian stimulation protocol for IVF. *Frontiers in Endocrinology*.

[10] Jang S., Kim K. H., Jun J. H., You S. (2020). Acupuncture for in vitro fertilization in women with poor ovarian response: a systematic review. *Integrative Medicine Research*.

[11] Lensen S. F., Wilkinson J., Leijdekkers J. A. (2018). Individualised gonadotropin dose selection using markers of ovarian reserve for women undergoing in vitro fertilisation plus intracytoplasmic sperm injection (IVF/ICSI). *Cochrane Database of Systematic Reviews*.

[12] Polyzos N. P., Tournaye H., Guzman L., Camus M., Nelson S. M. (2013). Predictors of ovarian response in women treated with corifollitropin alfa for in vitro fertilization/intracytoplasmic sperm injection. *Fertility and Sterility*.

[13] Oehninger S., Nelson S. M., Verweij P., Stegmann B. J. (2015). Predictive factors for ovarian response in a corifollitropin alfa/GnRH antagonist protocol for controlled ovarian stimulation in IVF/ICSI cycles. *Reproductive Biology and Endocrinology*.

[14] Zheng H., Chen S., Du H. (2017). Ovarian response prediction in controlled ovarian stimulation for IVF using anti-Müllerian hormone in Chinese women: a retrospective cohort study. *Medicine (Baltimore)*.

[15] Chen C. L. P., Liu Z. (2018). Broad learning system: an effective and efficient incremental learning system without the need for deep architecture. *IEEE Transactions on Neural Networks and Learning Systems*.

[16] Broer S. L., Dólleman M., Opmeer B. C., Fauser B. C., Mol B. W., Broekmans F. J. M. (2011). AMH and AFC as predictors of excessive response in controlled ovarian hyperstimulation: a meta-analysis. *Human Reproduction Update*.

[17] Delvigne A., Rozenberg S. (2002). Epidemiology and prevention of ovarian hyperstimulation syndrome (OHSS): a review. *Human Reproduction Update*.

[18] Aflatoonian A., Oskouian H., Ahmadi S., Oskouian L. (2009). Prediction of high ovarian response to controlled ovarian hyperstimulation: anti-Müllerian hormone versus small antral follicle count (2-6 mm). *Journal of Assisted Reproduction and Genetics*.

[19] Moolhuijsen L. M. E., Visser J. A. (2020). Anti-Müllerian hormone and ovarian reserve: update on assessing ovarian function. *The Journal of Clinical Endocrinology and Metabolism*.

[20] Pilsgaard F., Grynnerup A. G.-A., Løssl K., Bungum L., Pinborg A. (2018). The use of anti-Müllerian hormone for controlled ovarian stimulation in assisted reproductive technology, fertility assessment and -counseling. *Acta Obstetricia et Gynecologica Scandinavica*.

[21] Baker V. L., Gracia C., Glassner M. J. (2018). Multicenter evaluation of the access AMH antimullerian hormone assay for the prediction of antral follicle count and poor ovarian response to controlled ovarian stimulation. *Fertility and Sterility*.

[22] Iliodromiti S., Anderson R. A., Nelson S. M. (2015). Technical and performance characteristics of anti-Müllerian hormone and antral follicle count as biomarkers of ovarian response. *Human Reproduction Update*.

[23] Bruno-Gaston J., Jung J., Kumar T., Zarutskie P., Gibbons W., Devaraj S. (2021). Association of ovarian response with picoAMH in women undergoing controlled ovarian hyperstimulation. *Clinical Biochemistry*.

[24] Mohiyiddeen L., Newman W. G., McBurney H., Mulugeta B., Roberts S. A., Nardo L. G. (2012). Follicle-stimulating hormone receptor gene polymorphisms are not associated with ovarian reserve markers[J]. *Fertility and sterility*.

[25] Sun B., Ma Y., Li L. (2020). Factors associated with ovarian hyperstimulation syndrome (OHSS) severity in women with polycystic ovary syndrome undergoing IVF/ICSI. *Frontiers in Endocrinology*.

[26] Broekmans F. J., Verweij P. J. M., Eijkemans M. J. C., Mannaerts B. M. J. L., Witjes H. (2014). Prognostic models for high and low ovarian responses in controlled ovarian stimulation using a GnRH antagonist protocol. *Human Reproduction*.

[27] Mahran A., Khairy M., Elkhateeb R. (2021). The value of serum progesterone level on day of human chorionic gonadotrophin administration/metaphase II oocyte ratio in predicting IVF/ICSI outcome in patients with normal ovarian reserve. *Journal of Ovarian Research*.

[28] Requena A., Cruz M., Bosch E., Meseguer M., García-Velasco J. A. (2014). High progesterone levels in women with high ovarian response do not affect clinical outcomes: a retrospective cohort study. *Reproductive Biology and Endocrinology*.

[29] Xu B., Li Z., Zhang H. (2012). Serum progesterone level effects on the outcome of in vitro fertilization in patients with different ovarian response: an analysis of more than 10,000 cycles. *Fertility and Sterility*.

